# Risk miRNA screening of ovarian cancer based on miRNA functional synergistic network

This article has been retracted.

**DOI:** 10.1186/1757-2215-7-9

**Published:** 2014-01-21

**Authors:** Huanchun Ying, Jing Lyu, Tianshu Ying, Jun Li, Shanshan Jin, Jingru Shao, Lili Wang, Hongying Xu

**Affiliations:** 1 Department of Gynecology and Obstetrics, Shengjing Hospital of China Medical University, No.36, Sanhao Street, Heping District, Shenyang, Liaoning Province 110004, China; 2 Department of Oncology, the fifth Hospital of Shenyang, Shenyang 110023, China; 3 Department of Gynecology and Obstetrics, the ninth Hospital of Shenyang, Shenyang 110024, China

**Keywords:** miRNA expression profile, Ovarian cancer, miRNA functional synergistic network, Co-regulating, Functional module

## Abstract

**Background:**

miRNAs are proved to have causal roles in tumorgenesis involving various types of human cancers, but the mechanism is not clear. We aimed to explore the effect of miRNAs on the development of ovarian cancer and the underlying mechanism.

**Methods:**

The miRNA expression profile GSE31801 was downloaded from GEO (Gene Expression Omnibus) database. Firstly, the differentially expressed miRNAs were screened. Target genes of the miRNAs were collected from TargetScan, PicTar, miRanda, and DIANA-microT database, then the miRNA-miRNA co-regulating network was constructed using miRNA pairs with common regulated target genes. Next, the functional modules in the network were studied, the miRNA pairs regulated at least one modules were enriched to form the miRNA functional synergistic network (MFSN).

**Results:**

Risk miRNA were selected in MFSN according to the topological structure. Transcript factors (TFs) in MFSN were identified, followed by the miRNA-transcript factor networks construction. Totally, 42 up- and 61 down-regulated differentially expressed miRNAs were identified, of which 68 formed 2292 miRNA pairs in the miRNA-miRNA co-regulating network. GO: 0007268 (synaptic transmission) and GO: 0019226 (transmission of nerve impulse) were the two common functions of miRNAs in MFSN, and hsa-miR-579 (36), hsa-miR-942 (31), hsa-miR-105 (31), hsa-miR-150 (34), and hsa-miR-27a* (32) were selected as the hub nodes in MFSN.

**Conclusions:**

In all, 17 TFs, including CREM, ERG, and CREB1 were screened as the cancer related TFs in MFSN. Other TFs, such as BIN1, FOXN3, FOXK1, FOXP2, and ESRRG with high degrees may be inhibited in ovarian cancer. MFSN gave us a new shed light on the mechanism studies in ovarian cancer.

## Introduction

Ovarian cancer is a cancerous growth arising from the ovary, and a leading death from gynecologic malignancy in the western world, with a 5-year survival rate of approximately 30% in advanced-stage disease when diagnosed [1]. The vague and nonspecific symptoms, which usually appear when the patients has reached an advanced stage, have led to the high case-fatality ratio of ovarian cancer [2,3]. Thus, the molecular mechanism study on ovarian cancer is of great importance for women healthy.

MicroRNAs (miRNAs) control various cellular processes through the post-transcriptional regulatory network. The deregulation of miRNA is involved in the initiation and progression of human cancer [4], and the studies on ovarian cancer are widely conducted in the past few years. Zhang et al. [5] carried an integrative genomic approach for the identification of miRNA deregulation in human epithelial ovarian cancer. They found that miRNA expression was markedly down-regulated in malignant transformation and tumor progression, contributing to a genome-wide transcriptional deregulation. Resnick et al. [6] detected the differentially expressed microRNAs from the serum of ovarian cancer using a novel real-time PCR platform, and miRNAs-21, 92 and 93 were identified to be potential biomarkers. Oncogenic miRNA-27a is also found to be a therapeutic target for Ovarian cancer cells [7]. However, the potential mechanism and its contributions to genome-wide transcriptional changes in cancer are still remarkably unknown.

Synergistic regulations among multiple miRNAs are important to understand the mechanisms of complex post-transcriptional regulations in humans. Complex diseases, especially cancers are affected by several miRNAs rather than a single miRNA. Thus, it is a challenge to identify miRNA synergistic functions and thereby further determine miRNA functions at a system level and investigate disease miRNA features in the miRNA–miRNA synergistic network (MFSN) from a new view [8]. miRNA synergetic regulations are gradually identified by computational or experimental evidence. However, the potential characteristic underlying miRNA synergism remains a mystery [9].

In this study, we attempted to systematically dissect the risk miRNA of ovarian cancer, based on the constructed MFSN, from three levels: sequence, secondary structure and transcriptional regulation. Briefly, differentially expressed miRNAs were first identified, and then based on the correlations between miRNAs and target genes, miRNA-miRNA co-regulating network was constructed, and based on the functional cluster of the network, the MFSN was constructed. Next, the transcript factors (TFs) in MSFN were screened, the miRNA-transcript factors network was sequentially constructed.

## Materials and methods

### Affymetrix microarray analysis

We downloaded the miRNA expression profile data GSE31801 [10] from NCBI (National Center for Biotechnology Information) GEO (Gene Expression Omnibus) (http://www.ncbi.nlm.nih.gov/geo/) database. Chips of miRNA profiling in lymphoblastoid cell lines from 74 women with familial ovarian cancer were available, as well as chips from 47 normal ovarian tissues. The annotation information of the chip was also downloaded from GPL8179_humanMI_V2_R0_XS0000124_MAP platform.

### Data preprocessing

The original miRNA expression profile was first standardized using median method [11]. Then the probe level data were converted into miRNA names, and only one miRNA was chosen when there were more than one miRNAs responding to a signal probe.

### Differentially expressed miRNAs analysis

To screen the differentially expressed miRNAs, limma package in R language [12] was used, with the cut off criterion of adjusted p value less than 0.05, and |log fold change (FC)| larger than 1.5.

### miRNA-miRNA co-regulating network construction

TargetScan [13], PicTar [14], miRanda [15], and DIANA-microT [16] database was used to predict the target genes of miRNAs. Then the selected miRNAs-target genes database was used for the identification of the target genes of differentially expressed miRNAs. miRNA pairs having same regulating target genes were selected for the miRNA-miRNA co-regulating network construction using cytoscape software [17].

### Functional synergy analysis of differentially expressed miRNAs

For each miRNA pair, their co-regulating target genes was identified as a target subset, and then ClusterProfiler package [18] in R language was used to perform the candidate biological process (BP) functional modules identification. The threshold was set as p and q value less than 0.05. If a pair of miRNAs significantly co-regulated at least one functional module, the miRNAs were considered as synergistic miRNAs [8]. All the synergistic miRNA pairs were gathered to form a MFSN. Next, igraph package [19] was used to calculate the degrees of the nodes and the minimum radius of the MFSN. The numbers and the Gene Oncology (GO) BP terms of functional modules in MFSN were further analyzed.

### miRNA -transcription factor regulating network construction

We first identified the transcription factors (TFs) of the target genes in MFSN using TRANSFAC. Then we constructed the miRNA-transcription factor regulating network using the TFs and their interacted miRNAs. Finally, TRED database [20] was used to screen the verified cancer-related TFs in the network.

## Results

### Differentially expressed miRNAs

After preprocessing, we obtained the expression values of 1146 miRNAs of the 121 samples. In total, 42 up- and 61 down-regulated differentially expressed miRNAs were identified. There were 42411 and 55775 corresponding target genes of up- and down-regulated miRNAs respectively.

### miRNA-miRNA co-regulating network construction

The common regulated target genes of each miRNA pair were screened, and 2292 co-regulating pairs formed by a total of 68 miRNAs shared at least one target gene were screened, including 34 up-regulated miRNAs (Figure 1).

**Figure 1:** **Co-regulating network of differentially expressed miRNAs.** Red nodes represent up-regulated miRNAs, green nodes represent down-regulated miRNAs, and edges indicate that there are co-regulating target genes between the two miRNAs.

### MFSN network construction

GO terms enrichment of each miRNA pair in the co-regulating network was conducted, then, miRNA pairs regulating at least one functional module were collected to construct the MFSN network. There were 333 co-regulating pairs formed by 41 miRNAs (Figure 2) in the network, such as hsa-miR-342-5p, hsa-miR-628-3p, hsa-miR-600, and hsa-miR-647.

**Figure 2:** **Functional synergistic networks of differentially expressed miRNAs.** Red nodes are the up-regulated miRNAs, and the green nodes are the down-regulated miRNAs. Edges represent the synergistic effect between miRNAs.

Next, we discussed the structure and organization of the MFSN. The MFSN was a small word with a short diameter of 2, with a few miRNAs interacted with a relatively large number of miRNA partners, and many miRNAs have few miRNA partners. In all, 5 nodes with degrees more than 30, including hsa-miR-579 (36), hsa-miR-942 (31), hsa-miR-105 (31), hsa-miR-150 (34), and hsa-miR-27a* (32) were selected as the hub nodes in MFSN. Besides has-miR-579, the other four nodes were up-regulated differentially expressed miRNAs. Hub nodes with high degrees in MFSN have more close association with other miRNAs in function, thus are considered as risk miRNAs.

### Functional modules in MFSN analysis

The examination of number distribution of co-regulating functional modules revealed a power law tendency. In total, 73.3% miRNAs pairs (244) were involved in at least 5 modules (Figure 3), suggesting that these miRNAs participated cooperatively in many BPs in the development of ovarian, the up-/down-regulation of miRNAs would cause the dysfunctions of many BPs. The miRNA pair of hsa-miR-942 and hsa-miR-33a had the highest function module number of 279, and hsa-miR-942 as a hub node in MFSN, was synergistic with 31 miRNAs. Hsa-miR-942 was an up-regulated, while hsa-miR-33a was a down-regulated miRNAs in ovarian cancer.

**Figure 3:** **Distributions of function modules of synergistic miRNA pairs.** Horizontal axis represents the count of function module, while vertical axis represents the count of the miRNA pairs.

Next, we analyzed the distributions of GO BP terms enriched in MFSN. More than 85% miRNAs were enriched in the function module of GO: 0007268 (synaptic transmission) and GO: 0019226 (transmission of nerve impulse). As shown in Table 1 (the top 20 enriched functional modules), signal transduction related functions were the most frequent functions of the miRNAs in MFSN.

**Table 1:** Top 20 enriched biological process functions of the miRNA functional synergistic network

**Gene oncology (GO) biological process (BP) term & description**	**Percent**
GO:0007268 ~ synaptic transmission	0.867868
GO:0019226 ~ transmission of nerve impulse	0.864865
GO:0035637 ~ multicellular organismal signaling	0.855856
GO:0007267 ~ cell-cell signaling	0.651652
GO:0050877 ~ neurological system process	0.582583
GO:0003008 ~ system process	0.51952
GO:0007399 ~ nervous system development	0.474474
GO:0044700 ~ single organism signaling	0.447447
GO:0023052 ~ signaling	0.447447
GO:0007154 ~ cell communication	0.447447
GO:0030182 ~ neuron differentiation	0.444444
GO:0048666 ~ neuron development	0.435435
GO:0022008 ~ neurogenesis	0.432432
GO:0048731 ~ system development	0.42042
GO:0044707 ~ single-multicellular organism process	0.417417
GO:0048699 ~ generation of neurons	0.408408
GO:0007275 ~ multicellular organismal development	0.408408
GO:0031175 ~ neuron projection development	0.396396
GO:0048646 ~ anatomical structure formation involved in morphogenesis	0.381381
GO:0048812 ~ neuron projection morphogenesis	0.363363

### miRNA -transcription factor regulating network

Corresponding to the 2117 genes participated in the functional modules in MFSN, 90 TFs were identified. Then the miRNA-transcription factor regulating network was constructed (Figure 4). The TFs were mapped to TRED database, a total of 17 cancer related TFs coming from 13 TFs family were identified (Table 2). CREM, ERG, and CREB1 had the highest degrees among the 17 TFs, that is, 55, 38, and 28 respectively. They were collected for the construction of a new miRNA-transcription factor regulating network (Figure 5). In the rest 73 TFs among all the 90 target genes, BIN1 (26), FOXN3 (29), FOXK1 (31), FOXP2 (32), and ESRRG (42) were the top 5 TFs ranked by the numbers of miRNAs interacted with them.

**Figure 4:** **The regulating network of 17 cancer related transcript factors (TFs) and differentially expressed miRNAs.** Blue nodes are the TFs, red nodes are the up-regulated miRNAs, and green nodes are the down-regulated miRNAs. Edges represent the interactions between TFs and miRNAs.

**Table 2:** Cancer related transcript factors in the miRNA functional synergistic network

**Transcription factor**	**Family**	**Full name**	**Degree**
ARNT	HIF	Hypoxia-inducible factor	10
ATF3	ATF	Activating transcription factor	8
ATF7	ATF	Activating transcription factor	19
BCL6	BCL	B-cell CLL/lymphoma	3
BRCA2	BRCA	Breast cancer susceptibility protein	5
CREB1	CREB	cAMP responsive element binding protein	28
CREM	CREB	cAMP responsive element binding protein	55
E2F7	E2F	E2F transcription factor	14
EGR2	EGR	Early growth response protein	8
ELK1	ELK	Member of ETS oncogene family	5
ERG	ERG	ets-related gene	38
ESR2	ER	Estrogen receptor	3
ETS1	ETS	ETS-domain transcription factor	13
ETV4	ETS	ETS-domain transcription factor	3
FOSB	AP1	Activator protein 1	8
GLI3	GLI	Glioma-associated oncogene homolog	17
HIF1A	HIF	Hypoxia-inducible factor	7

**Figure 5:** **The regulating network of 3 main cancer related transcript factors (TFs) and differentially expressed miRNAs.** Blue nodes are the TFs, red nodes are the up-regulated miRNAs, and green nodes are the down-regulated miRNAs. Edges represent the interactions between TFs and miRNAs.

## Discussion

In order to obtain an in-depth analysis of individual miRNAs in the context of their synergistic surroundings, MFSN of differentially expressed miRNAs was constructed via co-regulating functional modules. Furthermore, the underlying functional patterns of risk miRNAs in ovarian cancer were also reported in this study. Among all the 103 differentially expressed miRNAs, 68 miRNAs formed 2292 pairs which shared at least one target genes. There were 41 miRNAs (333 miRNA pairs) in the miRNA-miRNA co-regulating shared at least one significant functional module. In addition, GO: 0007268 synaptic transmission and GO: 0019226 transmission of nerve impulse were the most common functional modules of miRNAs in MFSN. According to their degrees in MFSN, hsa-miR-579, hsa-miR-942, hsa-miR-105, hsa-miR-150, and hsa-miR-27a* were selected as hub nodes in MFSN. What’s more, 17 cancer-related TFs were identified in MFSN, which were further used for the miRNA-transcript factors network construction.

The selected 5 hub miRNAs in MFSN all had the degree more than 30, and they were considered as the potential ovarian cancer-related risk miRNAs, whose alternations were related to the dysfunctions of many BPs in ovarian cancer tissues. Hsa-miR-579 was a down-regulated miRNA of ovarian cancer samples, and miR-579 is found to dysregulated in colorectal cancer with liver metastasis [21]. The other four miRNAs, hsa-miR-942, hsa-miR-105, hsa-miR-150, and hsa-miR-27a* were identified to be up-regulated in ovarian cancer. The miRNA pairs comprised of hsa-miR-33a and hsa-miR-942 accounted for the richest functional module number of 279. There were 31 miRNAs interacted with hsa-miR-942 in MFSN, suggesting they were functionally synergistic with hsa-miR-942 and the expression changes of hsa-miR-942 in ovarian cancer may cause the changes of these connected miRNAs as well. The expression of miR-942 is significantly increased in patients with biliary tract cancer [22], and in late recurrent hepatocellular carcinoma samples [23]. In the formalin-fixed squamous cell carcinomas of the tongue, hsa-miR-105 is one of the up-regulated miRNAs [24], and highly expressed in seminoma [25]. Secreted monocytic miR-150 could enhance the targeted endothelial cell migration [26], and hsa-miR-150 is found to be differentially expressed in lung cancer tissues [27]. Hsa-miR-150 is recommended to be used as a circulating cancer marker [28]. In addition, hsa-miR-27a is reportedly down-regulated in many cancers, including breast and prostate cancer [29].

The common functional modules of miRNAs in MFSN were screened by calculating the GO BP terms distribution. It turned out that these miRNAs were mainly participated in signal transduction related functions, with synaptic transmission and transmission of nerve impulse as the most significant ones. Synaptic transmission is the process by which neurotransmitters are released, and bind to the receptors of another neuron. Nerve impulses are essential for the propagation of the signals [30]. The dysfunction of transmission of nerve impulse meant that the signal transmission was impaired in the development of ovarian cancer. The up-regulated genes in gliomas are associated with several processes, such as synaptic transmission and transmission of nerve impulse [31].

The transcriptional activator CREM (cAMP-responsive element-binding modulator) is highly expressed inpostmeiotic cells [32]. Down-regulated CREM modulates the transcription of several genes containing a cAMP responsive element motif in their promoter region [33]. CREM expression has been linked with several key physiological aspects of neuroendocrine pathways [34]. The aberrant expression of ERG (ETS transcription factor ) is demonstrated to be progression events in prostate tumorigenesis [35]. CREB1 (cAMP response element-binding protein 1) transduces cell survival responses to peptide hormones and growth factors in normal tissues, and mutant CREB proteins are implicated in tumorigenesis [36]. The TFs of CREM, ERG, and CREB1 were found to be regulated by several miRNAs in this study, which will influence the expressions of their target genes. The encoded genes by these TFs were potentially inhibited in ovarian cancer, as well as the regulations on the downstream target genes. What’s more, BIN1, FOXN3, FOXK1, FOXP2, and ESRRG were the top 5 TFs ranked by the numbers of miRNAs interacted with them, and their functions were inferred to be inhibited in ovarian cancer.

## Conclusion

In conclusion, risk miRNAs in ovarian cancer along with the interacted miRNAs can be detected by means of MFSN construction. The further study on the functional modules and TFs connection will provide a new approach on the mechanism study on miRNAs alternations in ovarian cancer.

## Competing interests

The authors declare that they have no competing interests.

## Authors’ contributions

HY and JL participated in the design of this study, and they both performed the statistical analysis. TY and JS carried out the study, and together with JL, LW collected important background information, and drafted the manuscript. SJ and HX conceived of this study, and participated in the design and helped to draft the manuscript. All authors read and approved the final manuscript.
